This article has been retracted.

# Efficacy of Electronic Cigarettes vs Varenicline and Nicotine Chewing Gum as an Aid to Stop Smoking: A Randomized Clinical Trial

**DOI:** 10.1001/jamainternmed.2023.7846

**Published:** 2024-01-29

**Authors:** Hao-Xiang Lin, Zhao Liu, Peter Hajek, Wan-Tong Zhang, Yuan Wu, Bao-Chen Zhu, Hai-Hua Liu, Qiu Xiang, Yan Zhang, Shu-Bin Li, Francesca Pesola, Ying-Ying Wang

**Affiliations:** 1 Institute for Global Health and Development, Peking University, Beijing, China; 2 Department of Tobacco Control and Prevention of Respiratory Disease, Center of Respiratory Medicine, China-Japan Friendship Hospital, Beijing, China; 3 Wolfson Institute of Population Health, Queen Mary University of London, London, England; 4 Institute of Clinical Pharmacology, Xiyuan Hospital, China Academy of Chinese Medical Sciences, Beijing, China; 5 China Academy of Chinese Medical Sciences, Beijing, China; 6 Department of Pharmacy, Dongzhimen Hospital, Beijing University of Chinese Medicine, Beijing, China; 7 Department of Traditional Chinese Medicine, Beijing Geriatric Hospital, Beijing, China; 8 Respiratory Intensive Care Unit, Tongji Hospital Affiliated with Tongji Medical College of Huazhong University of Science and Technology, Wuhan, China; 9 Office of China Journal of Traditional Chinese Medicine and Pharmacy, Beijing, China; 10 Beijing PL Technology Co, Ltd, Beijing, China; 11 Institute of Acupuncture and Moxibustion, China Academy of Chinese Medical Sciences, Beijing, China

## Abstract

**Importance:**

Electronic cigarettes (ECs) are often used by smokers as an aid to stopping smoking, but evidence is limited regarding their efficacy compared with nicotine replacement therapy (NRT), and no evidence is available on how their efficacy compares with that of varenicline.

**Objective:**

To evaluate whether ECs are superior to NRT and noninferior to varenicline in helping smokers quit.

**Design, Setting, and Participants:**

This was a randomized clinical trial conducted at 7 sites in China and including participants who were smoking at least 10 cigarettes per day and motivated to quit, not using stop-smoking medications or EC, and willing to use any of the study products. Participants were first recruited in May 2021, and data analysis was conducted in December 2022.

**Interventions:**

A cartridge-based EC (30 mg/mL nicotine salt for 2 weeks and 50 mg/mL after that), varenicline (0.5 mg, once a day for 3 days; 0.5 mg, twice a day for 4 days; and 1 mg, twice a day, after that), and 2 mg (for smokers of ≤20 cigarettes per day) or 4 mg (>20 cigarettes per day) nicotine chewing gum, all provided for 12 weeks and accompanied by minimal behavioral support (an invitation to join a self-help internet forum).

**Main Outcomes and Measures:**

The primary outcome was sustained abstinence from smoking at 6 months as validated by an expired-air carbon monoxide reading (<8 parts per million). Participants lost to follow-up were included as nonabstainers.

**Results:**

Of 1068 participants, 357 (33.5%) were female, and the mean (SD) age was 33.9 (3.1) years. A total of 409 (38.3%), 409 (38.3%), and 250 (23.4%) participants were randomized to the EC, varenicline, and NRT arms, respectively. The 6-month biochemically validated abstinence rates were 15.7% (n = 64), 14.2% (n = 58), and 8.8% (n = 22) in the EC, varenicline, and NRT study arms, respectively. The quit rate in the EC arm was noninferior to the varenicline arm (absolute risk reduction, 1.47%; 95% CI, −1.41% to 4.34%) and higher than in the NRT arm (odds ratio, 1.92; 95% CI, 1.15-3.21). Treatment adherence was similar in all study arms during the initial 3 months, but 257 participants (62.8%) in the EC arm were still using ECs at 6 months, with no further use in the 2 other study arms. The most common adverse reactions were throat irritation (32 [7.8%]) and mouth irritation (28 [6.9%]) in the EC arm, nausea (36 [8.8%]) in the varenicline arm, and throat irritation (20 [8.0%]) and mouth irritation (22 [8.8%]) in the NRT arm. No serious adverse events were recorded.

**Conclusions and Relevance:**

The results of this randomized clinical trial found that when all treatments were provided with minimal behavior support, the efficacy of EC was noninferior to varenicline and superior to nicotine chewing gum.

**Trial Registration:**

Chinese Clinical Trial Registry: ChiCTR2100048156

## Key Points

**Question:**

How do electronic cigarettes (ECs) as a stop-smoking aid compare with efficacy of varenicline and nicotine chewing gum?

**Findings:**

In this randomized clinical trial including 1068 smokers, ECs were as effective as varenicline and more effective than nicotine chewing gum when all 3 treatments were provided with minimal behavioral support.

**Meaning:**

ECs are an effective option for smokers seeking help with quitting smoking.

## Teaser

This randomized clinical trial examines whether electronic cigarettes are superior to nicotine replacement therapy and noninferior to varenicline in helping smokers quit.

## Introduction

The overall effects of electronic cigarettes (ECs) on public health remain disputed, with concerns about EC use in young people in contrast with the potential of ECs to help adult smokers quit.^1,2^ Regarding the function of ECs as an aid to stopping smoking, ECs can be seen as a form of nicotine replacement therapy (NRT) that is achieving a wider reach than traditional NRT products, such as nicotine chewing gum and nicotine patches. In countries where ECs and NRT are available, smokers tend to use ECs for smoking cessation more widely.^3,4^ Apart from the wider reach, a meta-analysis of 6 randomized clinical trials of ECs vs NRT conducted to date concluded that ECs were also more effective than NRT, although further trials are needed.^5^

Next to NRT, the most extensively tested and most widely used pharmacological aid to stopping smoking is a partial agonist for α4β2 nicotinic acetylcholine receptor, varenicline, which is also more effective than NRT.^6^ One study compared varenicline on its own with varenicline combined with ECs, but the trial was stopped early when only 46 participants were recruited in each study arm, meaning that the study was underpowered to detect a difference.^7^ To our knowledge, no study to date has attempted a direct comparison between ECs and varenicline.

In this article, we report a randomized clinical trial that compared ECs and varenicline. The trial also included an NRT arm. The trial was testing whether ECs are superior to NRT and noninferior to varenicline. The study was conducted in China, where access to and use of stop-smoking medications, as well as ECs, are much lower than in Western countries.^8,9,10,11,12^ This had the potential advantages of lower expectancy effects and reduced risk of trial arms contamination via use of nonallocated products, an issue that affected a recent UK trial of ECs vs NRT as treatments for pregnant smokers.^13^

## Methods

### Study Design

This was a multicenter, 3-arm, open-label, randomized clinical trial (Supplement 1). The trial was audited independently by China-Japan Friendship Hospital. The trial was approved by research ethics boards of participating centers.

### Participants

This study was conducted at 7 study sites: China-Japan Friendship Hospital (Beijing, China), Peking University Health Science Center (Beijing, China), Beijing Hospital (Beijing, China), Beijing Xiyuan Hospital (Beijing, China), Beijing Geriatric Hospital (Beijing, China), Beijing Dongzhimen Hospital (Beijing, China), and Wuhan Tongji Hospital (Wuhan, China). Participants were recruited via trial sites, local newspapers, community events, websites, and referrals from other medical institutions.

Participants were included if they smoked at least 10 cigarettes per day for at least 5 years, had expired air carbon monoxide (CO) reading of 9 parts per million (ppm) or greater, were age 25 to 45 years, and were motivated to stop smoking. Exclusion criteria included pregnancy or breastfeeding, use of stop-smoking medication during the previous 30 days, ever use of ECs for 7 days or longer, history of severe psychiatric illness, unwillingness to use study products, and current diagnosis of cancer or in remission from cancer for less than 1 year.

### Randomization and Masking

Randomization was conducted via a central randomization system for clinical research. Randomization sequences were generated using Proc Plan in SAS, version 9.3 (SAS Institute), with trial sites as the stratification factor and a block length of 5. After logging into the website, staff entered participants’ sex, age, and Fagerstrom Test for Cigarette Dependence (FTCD) score, and the system generated each participant’s identification number and treatment allocation via stratified block randomization. The study statistician was masked to treatment codes until the analysis of primary outcome was completed.

### Procedures

Potential participants contacted the local study sites to obtain study details and for eligibility checks. Eligible participants were invited for a baseline visit. At the visit, they provided a CO reading via a Bedfont Micro Smokerlyzer, their eligibility was confirmed, study details were discussed, and participants signed the informed consent form. They then filled in study questionnaires. After that, participants set up their target quit date (TQD), normally 2 weeks after the baseline visit.

Participants were then randomized into 1 of the 3 interventions and given their study product and instructions on how to use it. They were instructed to join a WeChat group for motivational support.

Finally, the date of the next visit 1 month later was agreed on, and participants received a $40 shopping voucher as compensation for their time and travel. The baseline visit took approximately 30 to 45 minutes.

Participants were then seen at the study center monthly for 6 months. At each visit, study forms were completed and CO readings were taken. Each follow-up visit took approximately 10 minutes.

During the study period, the products were provided free of charge. At the 3-month visit, participants were told that they could continue to use their products as needed, but would have to purchase them themselves. A leaflet was provided with information on where the products could be bought. At the last visit, participants received a $60 shopping voucher. The study started recruitment in May 2021 and completed all follow-ups in December 2022.

### Interventions

#### EC Arm

Participants received a cartridge-based EC product called RELX Wuxian (RELX Technology; eFigure 1 in Supplement 2) and a leaflet with product use instructions. The product was selected as it was easier to use than refillable EC and included a feature that delivered a warning buzz if users took more than 15 puffs in 15 minutes. The product was purchased from the manufacturers. Participants had a choice of 3 flavors with a nicotine salt concentration of 30 mg/mL: mung bean, watermelon, and ice cream (which were identified by retailers as the most popular flavors). Only 1 flavor, mint, was produced with a nicotine salt concentration of 50 mg/mL. Participants were instructed to use 30–mg/mL cartridges of their preferred flavor for the first 2 weeks and 50–mg/mL cartridges after that, but were asked to continue using 30 ng/mL or reverse to it if they did not like the higher strength. One cartridge was expected to last for 3 days. At the baseline session, 10 cartridges were provided, with an option to request additional supplies at 1-month and 2-month follow-ups (up to 30 cartridges altogether). Participants were instructed to start using their EC ad lib from the next day and stop smoking completely from their TQD onward.

#### Varenicline Arm

Participants received a 12-week supply of varenicline (Chantix; Pfizer) and a leaflet with product use instructions. Participants were instructed to take varenicline, 0.5 mg, once per day for the first 3 days, followed by 0.5 mg twice a day for the next 4 days and 1 mg twice a day from day 8, as per the *China Clinical Guidelines for Tobacco Cessation*.^14^ The product was purchased from the manufacturers. Participants were instructed to start using varenicline from the next day and stop smoking completely from their TQD onward.

#### NRT Arm

Participants received a 12-week supply of nicotine chewing gum (Johnson & Johnson) and a leaflet with product use instructions. Nicotine gum was selected as the most widely used form of NRT in China. Three boxes containing 105 pieces of the gum each were provided at each monthly contact, with an option to request additional supplies if needed. As specified by the China Clinical Smoking Cessation Guidelines^14^ and Chinese product labeling, participants who smoked up to 20 cigarettes per day (197 participants [78.8%] randomized into the NRT arm) received 2-mg nicotine gum, while those smoking 20 or more cigarettes per day (53 [21.2%]) received 4-mg nicotine gum. Both strengths were provided with the fresh mint flavor. Supplies were bought from the manufacturer. Participants were instructed to use 8 to 12 pieces per day during the first 6 weeks, 4 to 8 pieces per day during weeks 7 and 8, and 2 to 4 pieces per day during the final 4 weeks, as *per China Clinical Guidelines for Tobacco Cessation*.^14^ Participants were instructed to use their NRT from the next day and stop smoking completely from the TQD onward.

### Behavioral Support

Participants in all 3 study arms were invited to join a self-help forum set up for the trial participants on WeChat, a messaging app. This was to share their experience with stopping smoking and provide mutual support via text messages. WeChat was also used for scheduling study appointments and sending appointment reminders. No other behavioral support was provided.

### Measures

At baseline, demographic and smoking history variables were collected, including age, sex, ethnicity, education, marital status, income, health status, age of starting to smoke, cigarettes smoked per day, and previous cessation attempts. Participants also completed the FTCD,^15^ Hospital Anxiety and Depression Scale, ^16^ and Chronic Obstructive Pulmonary Disease (COPD) Assessment Test.^17^ Objective measures included weight, height, blood pressure, heart rate, and expired CO reading.

At each follow-up, participants provided information on their smoking status, ratings of withdrawal symptoms using the Minnesota Nicotine Withdrawal Scale,^18^ ratings of helpfulness of the allocated product in stopping smoking (on a 4-point scale from not at all helpful to very helpful), use of the allocated and nonallocated study products, and, in the EC arm, issues with EC product quality. Participants were also asked whether they experienced any of the following since the previous visit: abnormal dreams, restlessness, irritability, mouth ulcers, increased appetite, dry mouth, headache, weight gain, nausea, upper respiratory tract infection, constipation, hand tremor, fatigue, insomnia, dizziness, and difficulty concentrating. CO readings and weight were also collected and Hospital Anxiety and Depression Scale and COPD Assessment Test questionnaires were repeated. Blood pressure and heart rate were measured only at the 6-month session.

### Outcomes

The primary outcome was 6 months of sustained abstinence, defined as per the Russell standard^19^ as a self-report of smoking no more than 5 cigarettes from 2 weeks after the TQD and no smoking at all during the previous week, as validated by an expired CO level of less than 8 ppm at all points. Secondary abstinence outcomes comprised CO as validated by 7-day point-prevalence abstinence at each point. Participants lost to follow-up were included as nonabstainers. Treatment adherence outcomes included attendance at monthly sessions and self-reported use of allocated and nonallocated products. Other outcomes included ratings of treatments, monitoring of adverse reactions and recording of serious adverse events.

### Sample Size

In an earlier study of smokers with COPD in China, we recorded a 6-month quit rate with varenicline of 41.5% when varenicline was accompanied by intensive weekly support.^20^ A Cochrane review found higher quit rates when pharmacotherapy was accompanied by behavioral support vs pharmacotherapy without it (risk ratio [RR], 1.2).^21^ Thus, we estimated the quit rate with varenicline in this trial of around 35%. Regarding ECs, a previous large trial comparing ECs and NRT reported 6-month quit rates of 35.4% with refillable ECs with up to 18 mg/mL of nicotine.^22^ We estimated a similar quit rate in this trial, as it provided limited behavioral support but used a stronger nicotine liquid and more user-friendly vaping device. The quit rate in the NRT arm in the same study was 25.1%,^22^ achieved with combination NRT. Single NRT is less effective than combination NRT,^21^ and the lack of behavioral counseling can be expected to lower the quit rate as well, so we estimated the quit rate in the nicotine chewing gum group at 21%. To have a 90% probability of detecting the difference between 21% and 35% (*P* < .03, 2-tailed test), 250 participants were needed in each comparison group.

To test the noninferiority of ECs compared with varenicline, we selected the upper limit of 97.5% CIs of the difference between varenicline and ECs to include an absolute noninferiority margin of 10%. To have 85% power to detect this (α = .03, 1-tailed test), 409 participants were needed in each of the 2 study arms. In total, the trial aimed to recruit 409 + 409 + 250 participants, adding to 1068 participants.

### Statistical Analysis

Differences in baseline characteristics were assessed by analysis of variance for continuous variables and by χ^2^ test for categorical variables. For primary analyses, we used the intention-to-treat approach in which participants with unknown smoking status were included as nonabstainers so that all randomized participants were included.^19^ The study’s 2 primary objectives comprised a comparison of ECs vs NRT (expecting ECs to be more effective than NRT, as previously described) and a noninferiority comparison of ECs vs varenicline (using varenicline as the standard) in 6-month validated sustained abstinence rates. To adjust the calculations for 2 pairwise comparisons, an α of *P* = .03 was used for the sample size calculations and primary outcome analyses. Logistic regression analyses were used. In a sensitivity analysis, the model was adjusted for any baseline variables in which the study arms differed and for study sites. Secondary objectives included a comparison between varenicline and NRT and other abstinence and adherence outcomes listed previously. The results are presented as absolute risk reductions (ARRs) for noninferiority analyses and odds ratios (ORs) with 95% CI for superiority analyses. Statistical analyses were performed using SAS, version 9.4 (SAS Institute). Data were entered directly into an online database developed by Beijing PL Technology Co, Ltd.

## Results

Between May 2021 and June 2022, 1338 potential participants were screened, and 1068 eligible participants were randomly assigned to 1 of the 3 study arms (ECs: 409 [38.3%]; varenicline: 409 [38.3%]; NRT: 250 [23.4%]). Among participants randomized into the NRT arm, 197 (78.8%) who smoked up to 20 cigarettes per day received 2-mg nicotine gum, while 53 (21.2%) smoking 20 or more cigarettes per day received 4-mg nicotine gum. Altogether, 332 (81.2%), 330 (80.7%), and 200 participants (80.0%) in the EC, varenicline, and NRT arms, respectively, completed the 6-month follow-up (Figure). eFigure 2 in Supplement 2 shows the distribution of study dropouts over time.

**Figure.** Screening, Randomization, and Follow-Up

Baseline characteristics of the sample are shown in Table 1. Overall, there were 357 female participants (33.5%), the mean (SD) age was 33. 9 (3.1) years, and participants smoked on average 16 cigarettes per day.

**Table 1.** Baseline Characteristics

Baseline characteristic	No. (%)			
	EC (n = 409)	Varenicline (n = 409)	NRT (n = 250)	Total sample (N = 1068)
Sex				
Female	133 (32.5)	140 (34.2)	84 (33.7)	357 (33.5)
Male	276 (67.5)	269 (65.8)	166 (66.3)	711 (66.5)
Age, mean (SD), y	34.3 (3.2)	33.9 (3.2)	33.5 (3.0)	33.9 (3.1)
Ethnicity				
Han	382 (93.4)	388 (94.9)	234 (93.5)	1004 (94.0)
Other	27 (6.6)	21 (5.1)	16 (6.5)	64 (6.0)
Marital status				
Single	56 (13.7)	56 (13.8)	22 (8.7)	134 (12.5)
Married	346 (84.6)	342 (83.7)	224 (89.6)	912 (85.4)
Separated/divorced/widowed	7 (1.7)	11 (2.5)	4 (1.7)	22 (2.1)
Education				
Primary school	19 (4.8)	24 (5.9)	16 (6.2)	59 (5.5)
Middle and high school	153 (37.3)	148 (36.2)	112 (44.9)	413 (38.7)
College and higher education	237 (57.9)	237 (57.9)	122 (48.9)	596 (55.8)
Monthly income, ¥^a^				
<2999	77 (18.9)	63 (15.3)	40 (16.3)	180 (16.9)
3000-5999	147 (35.9)	163 (39.9)	104 (41.6)	414 (38.8)
6000-9999	115 (28.1)	112 (27.4)	65 (25.8)	292 (27.3)
>10 000	70 (17.1)	71 (17.4)	41 (16.3)	182 (17.0)
Self-reported health status				
Poor	82 (20.1)	79 (19.3)	46 (18.5)	207 (19.4)
Average	133 (32.5)	119 (29.1)	78 (31.2)	330 (30.9)
Good	194 (47.4)	211 (51.6)	126 (50.3)	531 (49.7)
CAT, mean (SD)	14.4 (9.9)	15.2 (9.2)	13.4 (6.5)	14.4 (8.9)
Blood pressure, mean (SD)				
Systolic, mm Hg	116.6 (13.4)	118.0 (14.1)	119.2 (12.9)	118.3 (13.3)
Diastolic, mm Hg	77.7 (10.5)	78.8 (10.5)	78.0 (10.5)	77.9 (9.4)
Current alcohol use				
Yes	241 (58.9)	255 (62.4)	150 (60.1)	646 (60.5)
No	168 (41.1)	154 (37.6)	100 (39.9)	422 (39.5)
BMI, mean (SD)	24.2 (3.4)	23.8 (3.6)	24.5 (3.3)	24.1 (3.2)
Chronic disease				
Yes	72 (17.6)	68 (16.6)	46 (18.5)	186 (17.4)
No	337 (82.4)	341 (83.4)	204 (81.5)	882 (82.6)
HADS score, mean (SD)	9.94 (5.7)	10.33 (7.2)	10.20 (7.5)	10.02 (7.0)
Cigarettes smoked per day, mean (SD)	16.8 (5.2)	15.7 (5.5)	15.6 (5.1)	16.0 (5.3)
Smoking duration, mean (SD), y	13.5 (3.9)	13.3 (3.7)	12.7 (3.6)	13.2 (3.8)
FTCD score (range, 0-10), mean (SD)	3.7 (1.8)	4.5 (2.3)	4.2 (2.2)	4.1 (2.1)
Previous quitting attempts				
Yes	214 (52.3)	198 (48.4)	126 (50.4)	538 (50.4)
Unaided	178 (83.2)	170 (85.9)	105 (83.3)	453 (84.2)
NRT	14 (6.5)	4 (2.0)	15 (11.9)	33 (6.1)
Varenicline	21 (9.8)	21 (10.6)	4 (3.2)	46 (8.6)
Other treatments	1 (0.5)	3 (1.5)	2 (1.6)	6 (1.1)
No	195 (47.7)	211 (51.6)	124 (49.6)	530 (49.6)

Abbreviations: BMI, body mass index (calculated as weight in kilograms divided by height in meters squared); CAT, Chronic Obstructive Pulmonary Disease Assessment Test; EC, electronic cigarettes; FTCD, Fagerstrom Test of Cigarette Dependence; HADS, Hospital Anxiety and Depression Scale; NRT, nicotine replacement treatment.

^a^ Exchange rate: 1 Chinese yuan = 0.14 USD.

The validated 6-month sustained abstinence rates were 15.7%, 14.2%, and 8.8% in the EC, varenicline, and NRT arms, respectively, with ECs noninferior to varenicline (ARR, 1.47%; 95% CI, −1.41% to 4.34%) and superior to NRT (OR, 1.92; 95% CI, 1.15-3.21; *P* = .001). The validated 7-day abstinence rates at 6 months were 30.3%, 27.9%, and 18.4% in the EC, varenicline, and NRT arm, respectively, with ECs noninferior to varenicline (ARR, 2.44%; 95% CI, −2.35% to 7.24%) and superior to NRT (OR, 2.20; 95% CI, 1.26-3.22; *P* < .001) on this outcome as well (Table 2; eFigures 3 and 4 in Supplement 2). Abstinence rates in the varenicline arm were significantly higher than those in the NRT arm in all comparisons (eTable 1 in Supplement 2).

**Table 2.** Validated Abstinence Rates at Different Points^a^

Outcome	No. (%)					EC vs varenicline	EC vs NRT
	EC (n = 409)		Varenicline (n = 409)	NRT (n = 250)		ARR (95% CI), %	OR (95% CI)
**Validated sustained abstinence** ^b^							
1 mo	108 (26.4)	113 (27.6)			44 (17.6)	−1.22 (−3.62 to 1.17)	1.68 (1.13 to 2.49)
2 mo	88 (21.5)	108 (26.4)			37 (14.8)	−4.89 (−14.47 to 4.69)	1.58 (1.04 to 2.41)
3 mo	79 (19.3)	89 (21.8)			28 (11.2)	−2.44 (−7.24 to 2.35)	1.90 (1.19 to 3.02)
4 mo	69 (16.9)	86 (21.0)			24 (9.6)	−4.16 (−12.30 to 3.99)	1.91 (1.17 to 3.13)
5 mo	65 (15.9)	71 (17.4)			22 (8.8)	−1.47 (−4.34 to 1.41)	1.96 (1.17 to 3.23)
6 mo^c^	64 (15.7)	58 (14.2)			22 (8.8)	1.47 (−1.41 to 4.34)	1.92 (1.15 to 3.21)
**Validated 7-d point abstinence** ^d^							
1 mo	142 (34.7)	151 (36.9)			59 (23.6)	−2.20 (−6.51 to 2.11)	1.89 (1.36 to 2.40)
2 mo	151 (36.9)	168 (41.1)			68 (27.2)	−4.16 (−12.30 to 3.99)	1.88 (1.37 to 2.58)
3 mo	157 (38.4)	182 (44.5)			77 (30.8)	−6.11 (−18.09 to 5.87)	1.46 (1.04 to 2.05)
4 mo	138 (33.7)	122 (29.8)			63 (25.2)	3.91 (−3.76 to 11.58)	1.92 (1.36 to 2.70)
5 mo	132 (32.3)	118 (28.9)			58 (23.2)	3.42 (−3.29 to 10.13)	2.02 (1.43 to 2.86)
6 mo	124 (30.3)	114 (27.9)			46 (18.4)	2.44 (−2.35 to 7.24)	2.20 (1.26 to 3.22)

Abbreviations: ARR, absolute risk reductions; CO, carbon monoxide; EC, electronic cigarettes; OR, odds ratio; NRT, nicotine replacement treatment; ppm, parts per million; TQD, target quit date.

^a^ CO less than 8 ppm.

^b^ Validated sustained abstinence was defined as a self-report of smoking no more than 5 cigarettes from 2 weeks after the TQD and no smoking at all during the previous week, as validated by an expired CO level of less than 8 ppm at all points.

^c^ Primary outcome.

^d^ Validated 7-day point-prevalence abstinence was defined as a self-report of no smoking during the previous week, as validated by an expired CO level of less than 8 ppm.

As the study arms differed in education level and FTCD scores at baseline, we conducted a sensitivity analysis that controlled for these 2 variables as well as study sites. The results remained unchanged (EC vs varenicline: ARR, 1.47%; 95% CI, −1.41% to 4.34%; EC vs NRT: adjusted OR, 1.89; 95% CI, 1.13-3.17; varenicline vs NRT: adjusted OR, 1.82; 95% CI, 1.07-3.08; eTable 3 in Supplement 2). Self-reported abstinence rates showed the same pattern as validated quit rates in unadjusted and adjusted analyses (eTables 3 and 4 in Supplement 2).

Treatment adherence was similar in the 3 study arms during the first 3 months (Figure and Table 3). During the second 3 months, product use continued in the EC arm only, with 314 (76.8%), 285 (69.7%), and 255 (62.3%) EC arm participants using ECs at 4, 5, and 6 months, respectively. Among abstainers at 6 months in the EC arm, 43 of 64 (67.2%) were using ECs. No use of any of the study products was recorded in the varenicline and NRT arms after the initial 3 months. Ratings of helpfulness of the products in assisting participants in stopping smoking mirrored the efficacy outcomes, with NRT rated as less helpful than ECs and varenicline, and EC and varenicline rated as similarly helpful (eTable 5 in Supplement 2).

**Table 3.** Treatment Adherence

Treatment adherence	No. (%)				
	EC (n = 409)		Varenicline (n = 409)	NRT (n = 250)	
Set TQD	409 (100.0)	409 (100.0)			250 (100.0)
Used at least 1 dose of treatment	409 (100.0)	409 (100.0)			250 (100.0)
Using allocated treatment at 3-mo follow-up	342 (83.6)	352 (86.1)			200 (80.0)
Using allocated treatment at 6-mo follow-up	257 (62.8)	0			0
Used nonallocated treatment at any point	0	0			0

Abbreviations: EC, electronic cigarettes; NRT, nicotine replacement treatment; TQD, target quit date.

Adverse reactions were infrequent and included primarily throat and mouth irritation in the EC and NRT arms and nausea in the varenicline arm. No serious adverse events were reported in any of the 3 study arms (Table 4).

**Table 4.** Adverse Reactions and Serious Adverse Events

Variables, No. (%)	No. (%)		
	EC (n = 409)	Varenicline (n = 409)	NRT (n = 250)
**Adverse reactions** ^a^			
Throat irritation	32 (7.8)	0	20 (8.0)
Mouth irritation	28 (6.9)	1 (0.2)	22 (8.8)
Dry cough	2 (5.4)	5 (1.2)	4 (1.6)
Headache	2 (0.5)	9 (2.2)	8 (3.2)
Poor sleep	5 (1.2)	15 (3.7)	13 (5.2)
Nausea	0	36 (8.8)	13 (3.2)
Others	6 (1.5)	14 (3.4)	4 (1.6)
No. reporting at least 1 adverse reaction	37 (9.0)	41 (10.0)	25 (10.0)
**Serious adverse events**	0	0	0

Abbreviations: EC, electronic cigarettes; NRT, nicotine replacement treatment.

^a^ Number of participants who reported the reaction on at least 1 occasion.

## Discussion

In this randomized clinical trial, ECs were as effective in helping smokers quit as varenicline and more effective than nicotine chewing gum when all 3 products were provided with minimal behavioral support. The finding that ECs were superior to NRT in helping smokers quit aligns with previous studies. The effect size in this trial (RR, 1.78) is somewhat higher than that in the combined previous trials (RR, 1.63),^5^ which could be because this was to our knowledge the first trial that included an EC product using nicotine salt with a higher nicotine content. In addition, while in some countries, including China, product labeling and local guidelines recommend 4-mg gum to those smoking 20 or more cigarettes per day, in other countries, 4-mg gum is recommended to those smoking within 30 minutes of waking up. The first approach may result in fewer smokers using the higher-strength product, which could lower NRT efficacy. The trial used a single NRT product as a comparator. A combination of NRT products is more effective than single NRT,^23^ and a trial that compared ECs with combination NRT reported a lower effect size at 6 months^22^ (RR, 1.36; 95% CI, 1.15- 2.6.9) than found in the current study. The finding that EC had similar efficacy to varenicline corresponded with a previous finding showing varenicline as superior to NRT, with a difference in efficacy similar to that found between EC and NRT.^24^

As in previous studies, a much higher proportion of participants in the EC arm than in the other arms continued to use their product throughout the study period (63% vs 0%). The key question about long-term switching from smoking to EC use is whether this is a positive or a negative outcome. Extended EC use may be beneficial for some previous smokers by helping them to maintain some of the subjective rewards of smoking, avoid postcessation weight gain, or prevent relapse. However, although EC use is expected to pose few health risks of smoking, some adverse health outcomes of long-term EC use are likely.^25,26^ Varenicline is not used long term and so has an advantage in this respect.

Adverse reactions to all 3 products were infrequent and minor. For ECs, these included mouth and throat irritation and dry cough, affecting 7% to 8% of users; for nicotine chewing gum, it was mouth and throat irritation and poor sleep (5%-9%), and for varenicline, nausea (9%). As in previous studies, no major risks of EC use emerged over the relatively brief study period.

### Limitations

The trial had several limitations. The results may have been affected by several external events. In May 2021, the China Health Commission (equivalent to Ministry of Health) published *China’s Report on the Health Hazards of Smoking 2020,*^26^ which concluded that EC use is unsafe. This conclusion was widely reported by Chinese media during the next year or so and discussed repeatedly at the WeChat forum, and we estimate that it led some 20% of participants in the EC arm to stop EC use. In August 2021, Pfizer recalled varenicline because levels of N-nitroso-varenicline were found to be greater than the US Food and Drug Administration safety threshold.^27^ We notified the ethics committee, and the committee approved study continuation but requested that study participants be notified of the possible risks of N-nitroso-varenicline. As a result, we estimate that some 15% of participants in the varenicline arm stopped using their product. These events may have reduced quit rates in the EC and varenicline arms, but this would dilute rather than amplify the difference between these 2 arms and the NRT arm. Another external event affecting the trial was the COVID-19 pandemic. The lockdowns made the collection of CO readings difficult, particularly during 2 periods in 2022 shown in eFigure 2 in Supplement 2 when most study dropouts were recorded. This reduced the validated quit rates, but all 3 study arms were affected equally. This cluster of events is the likely reason for quit rates being lower than expected in our power calculations. Validated 7-day point prevalence abstinence rates were affected less, and effect sizes for all outcomes were close to those predicted, but the lower quit rates have reduced the statistical power for the primary outcome. Another key limitation of open-label trials is that participants’ expectations can affect outcomes. In smoking cessation studies, the results can be biased if participants randomized to what they perceive as an inferior option are less likely to use their treatment or are more likely to drop out of the trial. We tried to minimize this risk by only including participants who were willing to use any of the study products. Expectations may be also less of a problem among smokers in China, where stop-smoking medications and EC are much less popular than among smokers in the West.^8,9,10,11,12^ Indeed, 92% of trial participants had no previous experience with any stop-smoking treatment. Regarding adherence, all study participants set their TQD and all initiated their treatment. Product use during the initial 3-month study period was also similar in all 3 study arms, and relatively high. Dropout rates were almost identical in all 3 study arms. These findings are reassuring in that they suggest that the study results were unlikely to be affected by expectations.

Another potential risk in studies of this type is the use of nonallocated products. In a recent large trial comparing NRT and EC in pregnant smokers, a proportion of participants randomized to NRT stopped smoking successfully with the help of EC, making the unadjusted results difficult to interpret.^13^ The current trial benefited from the limited popularity of study products in China in this respect as well, as no self-reported use of nonallocated products was detected.

Due to concerns about adverse events being more likely in older age groups, the sample was limited to adults aged 25 to 45 years. Caution is needed in generalizing the results to older smokers.

Previous trials that compared ECs and NRT mostly complemented these treatments with intensive behavioral support.^5^ This raises an important question of whether ECs are effective without such clinical involvement. The present trial suggests that they are, but it does not provide a definitive answer. Although only minimal behavioral support was included, smokers were still asked to set up a TQD and their smoking status was checked monthly, features that are not available to smokers using ECs on their own. To see whether public health messages on EC use for smoking cessation need to include advice to use any additional support, further studies are needed that compare effects of different levels of behavioral support added to ECs.

The current trial results may help to clarify another question concerning previous trials. Most participants in stop-smoking trials in the West have previous experience with stop-smoking medications. For example, in a previous large trial comparing EC and NRT conducted within the stop-smoking services in the UK,^13^ 75% of the participants had tried treatment with NRT in the past. This raises a concern that the results of EC comparisons with other treatments may apply only to smokers who did not experience results with the alternative treatments in the past. This study replicated the previous findings of ECs being more effective than NRT despite only 3% of participants having had tried treatment with NRT before.

## Conclusions

In this randomized clinical trial that included participants with little previous experience of stop-smoking treatments and that provided only minimal behavioral support, ECs were as effective as varenicline and more effective than nicotine chewing gum as an aid in quitting smoking. As 63% of participants in the EC arm still used their products at 6 months, further studies are needed to assess whether such use is beneficial or harmful.

## Notes

Supplement 1. Trial protocol

Supplement 2. eFigure 1. E-cigarette product used in the study eFigure 2. Number of participants dropping out of the trial at each month eFigure 3. Validated sustained abstinence rates over time eFigure 4. Validated 7-days abstinence rates over time eTable 1. Unadjusted differences between varenicline and NRT in validated abstinence rates eTable 2. Unadjusted self-reported abstinence rates at different time points eTable 3. Adjusted differences in validated abstinence rates at different time points eTable 4. Adjusted differences in self-reported abstinence rates eTable 5. Ratings of product helpfulness at 3 and at 6 months

Supplement 3. Data sharing statement
